# Impact of Sociocultural Factors on Contraceptive Use: A Case Study of Pakistan

**DOI:** 10.1155/2022/2939166

**Published:** 2022-09-14

**Authors:** Arsalan Khan, Moiz Qureshi, Muhammad Daniyal, Kassim Tawiah

**Affiliations:** ^1^Department of Statistics, Quaid-i-Azam University, Islamabad, Pakistan; ^2^Department of Statistics, Shaheed Benazir Bhutto University, Shaheed Benazirabad, Pakistan; ^3^Department of Statistics, Islamia University of Bahawalpur, Pakistan; ^4^Department of Mathematics and Statistics, University of Energy and Natural Resources, Sunyani, Ghana; ^5^Department of Statistics and Actuarial Science, Kwame Nkrumah University of Science and Technology, Kumasi, Ghana

## Abstract

**Background:**

The use of birth control methods is influenced by complex and competing socioeconomic and demographic factors. Regardless of the complexity of the behavioral approach of women, the utility of contraceptive methods in providing the opportunity of choice is well paired. This study examined the factors driving the usage of contraception and the impact of contraceptive practices on population growth in Pakistan. We also perused the quantification of sociocultural contraceptive use. *Methodology.* The Pakistan Demographic and Health Survey (PDHS, 2017-18) dataset collected by the National Institute of Population Study (NIPS) was used for all analyses. We applied the frequentist logistic regression model and multinomial logistic regression model in assessing factors impacting contraceptive practices. Bayesian logistic and multinomial regression models were also implemented to compare estimates. The regions and provinces in Pakistan were considered as different clusters, thereby introducing hierarchical structures in the regression model.

**Results:**

The study revealed a distinctive highly significant negative effect on contraceptive use and women's age. The odds ratio (OR) for women aged 25-34, 35-44, and above 44 was 1.242, 1.155, and 0.638, respectively, which shows that the OR of contraceptive use decreases in women aged 25-44. Our study showed the superior performance of the Bayesian model in highlighting disparities among the various cultural streams existing in the country. Estimates of the Bayesian analysis of competing models indicated that the Bayesian models provide powerful estimates compared to the classical models.

**Conclusion:**

Our results indicated that contraceptive use is almost relevant to sociodemographic factors (education, age, language, partner, work, etc.). Women with no formal education living in rural areas were not aware of the use of contraception, thereby not using it. Contraceptive use and methods are most probably influenced by the age and the number of children of women. We recommend that high-quality education, counseling, and widespread access to contraceptives should be prioritized in family planning healthcare in all areas of the country, especially rural areas.

## 1. Introduction

The world's population grew slowly from 1.0 billion in 1800 to 2.5 billion in 1950. The growth in the population has accelerated, although slowly, to over 7.0 billion in recent times [1]. The United Nations (UN) expects this figure to grow to 9.1 billion in 2050 [2]. The absolute increments in the world population size remain large, about 75 million a year [3, 4].

Demographic and Health Surveys (DHS) are national representative household surveys that have been conducted since 1984 in more than 85 countries [5]. The DHS is designed to explore demographic, family planning, and fertility data collected in the Contraceptive Prevalence Surveys (CPS) and World Fertility Surveys (WFS) to provide a necessary resource for monitoring and evaluation of vital statistics and health indicators in developing countries. The DHS data spans on a wide range of objectives with a focus on fertility indicators, maternal and child health, reproductive health, nutrition, mortality, and health behavior in adults. The main advantages of DHS are high response rates, employment of qualified and trained interviewers, national coverage, worldwide, standardized data collection procedures, and consistent material over time, comparable across populations cross-sectionally as well as over time. In Pakistan, the National Center of Population study (NIPS), Islamabad, conducts the Pakistan DHS (PDHS) in collaboration with the National Center of Population Study (NCPS).

Contraceptive prevalence rate varies dramatically worldwide from one region to another. In Latin America and the Caribbean, the rate stands at 51%, while in Middle East and West Africa, the rate is 9% [6]. Westoff [6] showed that among average married women, 11% use traditional contraception while 32% practice modern contraceptive methods. For fertile women of childbearing age to prevent pregnancy, their behavior and consciousness may help them to do so by using contraception [7, 8].

Globally, rates of contraception usage are variable, with the UN reporting an average of 64% of married or in-union women of reproductive age using some form of contraception. The rate is the highest (75%) in North America and the lowest (33%) in Africa [9]. The advertent rates of pregnancy (PRs) of 52 per 1,000 reproductive-age women in the United State of America in 2006 was seen to be highly compared with many other industrialized countries, and about half of all pregnancies are unplanned [10]. The most common contraceptive methods used by women around the world at the time of this study are pill which is 28% (10.6 million) women and female sterilization 27% (10.2 million) women [11].

Pakistan is projected to be among the most populated countries by 2050 [2]. The country's population is approximately 21 million [2]. It is the fifth largest country in the world. Pakistan is currently having a clear disparity in population needs and available facilities [2]. Najmi et al. [12] proved that birth control usage increased from 11.9% in 1990 to 35% in 2013 with the fertility rate declining from 5.4 births per woman in 1990 to 3.7 in 2019. They argued that previous contraceptive use has prevented an estimated 43.8 maternal deaths per 100,000 live births yearly, amounting to 260,000 reductions in maternal deaths yearly [9, 13].

Contraceptive use is influenced by the multitude of factors. It plays an important role in family planning. There is a widely accepted association between contraceptive prevalence rate and total fertility rate [14], which motivates extensive demographic research in developing countries. Davidson et al. [15] proved that family planning attitudes and behavior among Somali and Eritrean refugees are highly affected by culture, religion, and refugee status. Agyei and Migadde [16] opined that sociocultural and demographic factors highly influence contraceptive knowledge, attitudes, and practices.

Folkloric contraceptive methods are very prevalent in Pakistan [17]. Folkloric contraceptives refers to local and spiritual methods of unproven effectiveness, for example, amulets, herbs, and beads. According to the 2012–2013 PDHS, the prevalence of sexually active fertile women who do not use contraception was 46%, with about 37% of these women residing in urban areas and 53% in rural areas [18]. Many potential barriers exist to contraceptive use among women of reproductive age (WRA) in Pakistan, such as the social, cultural, and perceived religious unacceptability of contraception, lack of knowledge and awareness of contraception, cost of contraceptives, and access to contraceptive services [19–22].

This paper highlights the impact of socioeconomic and cultural factors on birth control methods and contraceptive use as well as contraceptive prevalence in Pakistan from multistage clustered 2017-18 PDHS data. We investigated factors affecting the regulation of fertility through contraception in the context of classical and Bayesian logistic and multinomial modeling by measuring the influence of the combination of selected sociocultural and socioeconomic factors on the current contraceptive practice of women in Pakistan. We also examined the preference for contraceptive methods among women aged 15-49. The study will enable the Government of Pakistan to embark on targeted campaigns to sensitize women of all ages to the use and importance of contraceptives in the country.

The rest of the paper describes the data used, the methods applied in the analysis, the results of the analysis, and its discussion vis-a-vis the conclusion of the study.

## 2. Materials and Methods

### 2.1. Data

We explored data from the 2017-18 PDHS which is arguably the best available source of information on Pakistan contraceptive use. The PDHS surveyed males and females, but our analyses were limited to female respondents because their responses to questions about contraceptive use are considered more accurate. We previously published estimates using a partial version of this dataset, the 2012-13 PDHS [18]. This earlier version contained data from interviews with 44600 women. In this article, we present estimates for the current period spanning 2017-18. The NIPS in Islamabad conducted the survey to obtain the dataset after which it was made public.  Figure 1 is an illustration of a multiple bar graph reflecting the contraceptive use across the varying ages of women. The graph shows that the usage of contraception is high in women aged 25-44, which is reasonable because they are among the most fertile group of women [2]. The 2011-13 National Survey of Population Growth (NSPG) [23] showed that 67.4% of women aged 25-34 use contraceptives while 70% of those aged 35-44 use them. For women aged 15-24, it emerged that only 47.7% use contraceptives. This relation is also checked for urban and rural areas and provinces of Pakistan in Figure 2 with different representations. One can infer from the graph that contraceptive usage among women is similar in all rural areas as well as all urban areas. Detailed variable descriptions are presented in Table 1 in the appendix.

### 2.2. Methods

After the completion of hectic work on the collection of survey data related to birth control methods, the PDHS reports provided only cell frequency tabulation and visual display of the relationship between contraceptive use (women using birth control methods or not) and other socioeconomic and demographic factors such as region, education, marital matatus, wealth index, and age without any valid statistical estimation of parameters and confidence intervals for women across regions, provinces, rural, and urban areas. Based on the rigorous estimation, one can also develop regression models for contraception. Thus, to better articulate a more applicable form of the data, we explored the classical logistic regression model [24] and multinomial logistic regression model [6] on it. We also provided Bayesian logistic and multinomial regression models [25] to compare estimates.

#### 2.2.1. Classical Logistic Regression

This type of statistical model (also known as the logit model) is often used for classification and predictive analysis. Logistic regression estimates the probability of an event occurring, such as using a contraceptive or not using a contraceptive, based on a given dataset of independent variables [24]. One of the important assumptions of the linear regression model is that the error term of the model follows a normal distribution. Sometimes, the assumptions meet through the transformation of the response variable when a continuous response variable is skewed. However, when the response variable is categorical or discrete, a simple transformation cannot produce normally distributed residual errors. In such situations, generalized linear models (GLMs) in which the response variables of interest, such as “Yes”/“No” responses, do not have a full range (i.e., *−∞* to +*∞*) are recommended. In our case, we have a response of the form

(1) $$\begin{array}{c} y_{i}=\left\{\begin{array}{cc} 1, & \text{using birth control methods},\\ 0, & \text{otherwise}. \end{array}\right. \end{array}$$

The classical logistic regression analysis extends the technique of multiple regression analysis to study the situation in which the response is categorical. In practice, situations involving categorical outcomes are quite common. In our study, the response variable (contraceptive use) is categorical and has two outcomes ever married women or union women using contraception or not. The logistic regression is used to evaluate the effect of socioeconomic and demographic factors on birth control methods. The logistic regression model is of the form

(2) $$\begin{array}{c} \mathrm{Pr}\left[y_{i}=1\right]={\text{logit}}^{-1}\left(\alpha_{i}+\beta^{\text{age}}{\text{age}}_{i}+\beta^{\text{region}}{\text{region}}_{i}+\beta^{\text{province}}{\text{province}}_{i}+\beta^{\text{education}}{\text{education}}_{i}+\beta^{\text{language}}{\text{language}}_{i}+\beta^{\text{children}}{\text{children}}_{i}+\beta^{\text{work}}{\text{work}}_{i}+\beta^{\text{wealth}}{\text{wealth}}_{i}\right)\text{ for }i=1,\cdots ,n_{i}, \end{array}$$

where *α*_*i*_ is the intercept, and the *β*′*s* represent the coefficient of the independent variables.

#### 2.2.2. Classical Multinomial Logistic Regression

Multinomial logistic regression is used to predict the probability of a category of members on a response variable based on multiple independent variables. The classical multinomial logistic regression is applied when we have more than two categories in the response variable [6]. The response variable has three categories in our case, i.e., sterilization, traditional, and modern methods of birth control. The multinomial logistic regression in our study is of the form

(3) $$\begin{array}{c} \text{logit}\left(y_{i}=1\right)=\log\left(\frac{\delta_{i}}{1-\delta_{i}}\right)=\alpha_{i}+\beta^{\text{age}}{\text{age}}_{i}+\beta^{\text{region}}{\text{region}}_{i}+\beta^{\text{province}}{\text{province}}_{i}+\beta^{\text{education}}{\text{education}}_{i}+\beta^{\text{language}}{\text{language}}_{i}+\beta^{\text{children}}{\text{children}}_{i}+\beta^{\text{work}}{\text{work}}_{i}+\beta^{\text{wealth}}{\text{wealth}}_{i}\text{for }i=1,\cdots ,n_{i}, \end{array}$$

where *δ*_*i*_ is the probability of using the  *i* − th birth control method, *α*_*i*_ is the intercept, and the *β*′*s* represent the coefficient of the independent variables

(4) $$\begin{array}{c} y_{i}=\left\{\begin{array}{cc} 2, & \text{would take a sterilization},\\ 3, & \text{using the traditional methods},\\ 4, & \text{using modern method}. \end{array}\right. \end{array}$$

“2” is if the women would like to prefer sterilization, “3” is for women using the traditional methods, and “4” is for women who take modern methods.

#### 2.2.3. Bayesian Framework

One of the most important academic debates in which statisticians participated is the argument of using the classical and Bayesian methods of statistical analysis. Instead of instinctively jumping to one side, both methods of research should be learned and implemented where they seem necessary. In this way, Bayesian methods of estimation and inference have recently been used extensively. We cannot make a probability assumption explicitly on the parameters involved in the parent distribution in classical inference. A *p* value should not be interpreted as the likelihood that the null hypothesis is true, but instead refers to the probability that the data will be observed or even more extreme than when the null hypothesis is true. The likelihood of the values of parameters can be directly obtained in the Bayesian inference by finding, at the right of the region of that value, the area of the posterior distribution, which is equal to the proportion of the values of the parameter in the posterior sample larger than that value [25]. We may use this data to file the results of Bayesian statistical analysis as a means of estimating parameters with so-called 95% Bayesian credible intervals.

In the Bayesian viewpoint [25], we formulate linear regression using probability distributions rather than point estimates. In this paper, we use the Bayesian regression model to predict the outcome of the nonsampled set [26, 27]. What we obtain from frequentist linear regression is an estimation of model parameters from the training data set individually (the sampled data set in our problem). The sampled data informs our model entirely: in this sense, all that we need to identify is the model available in the sampled data. However, if the sample size is small, the estimate could be expressed as a distribution of possible parameter values given the sample details, which calls for the need of the Bayesian regression model. We were much concerned with programming errors in the Bayesian model fitting involving Markov Chain Monte Carlo (MCMC) as well as the problems that occur in its estimation procedures [28–30]. The trade-off with this extra task is that there is large flexibility in model construction, statistical inference, and assessment of model fit than the frequentist test.

Aside from these basic programming errors that can make the MCMC algorithm inadequate, there are two main concerns with the employment of the MCMC algorithm: mixing and convergence [31]. We confirmed that the algorithm results in the Markov chain, converges to the appropriate posterior density, and mixes well throughout the values of the density. We implemented the Bayesian logistic regression model by adding a normal before the coefficient of the linear log-mean function as in *β*_*i*_ ~ *N*(0, 1 × *e*^−3^) for all *i* = 0, 1, 2, ⋯, 25 [32]. The analysis is done on rjags in *R* using Just Another Gibbs Sampler (JAGS) taking three chains [33–35]. We initialize the model and run the burn-in period. The model is updated 150 times, and the number of iterations is taken to be 10000. A more reliable estimate for burn-in cut-off is through the effective sample size (ESS). An ESS is the number of independent samples that are equivalent to the number of autocorrelated samples. The burn-in can contain samples that do not have much information, thereby reducing the effective sample size (ESS) if the period of burn-in is predicted to be small enough [33–35]. Again, the much longer predicted burn-in is the cause of the small ESS as informative samples are being segregated. Practical estimation techniques strongly recommend an increase in ESS to the optimum approximation of the burn-in. We evaluated the burn-in samples at a glance by the ESS and trace plots.

## 3. Results and Discussion

### 3.1. Classical Logistic and Multinomial Logistic Regression

Table 2 provides the estimation from the logistic regression for contraceptive indicators with independent variables. In addition to the estimates of the model for the contraceptive indicators, the table provides standard errors (SE), odds ratio (OR), lower and upper bounds of the confidence interval, and *p* values. Table 2 reveals the effect of the independent variables on contraception. There was a distinctive highly significant negative effect of women's age on contraception with odds ratio (OR) 1.242, 1.155, and 0.638 for women aged 25-34, 35-44, and above 44, respectively. This shows a decreasing OR in the usage of contraception as the age of women increases above the 15-24 age group. We observed that women from rural areas are less likely to use birth control methods than their counterparts in urban areas. Similarly, the language was observed to have a highly significant effect on the likes of Baluchi, Sindhi, Saraiki, and other Urdu languages. However, Punjabi and Pushto speakers were not significant.

From Table 3, we see that birth control usage in urban areas and the corresponding language factor in urban areas are highly significant compared to rural areas. The insignificant effect of Islamabad for both areas (rural and urban) compared to Punjab shows that the contraceptive behavior is similar in both Punjab and Islamabad territory.

Table 4 provides contraceptive use for six different regions (four provinces, ICT, and FATA) including Gilgit-Baltistan and Azad, Jammu, and Kashmir (AJK) by using the separate logistic regression model. The tables present estimates of parameters, standard errors (SEs), and OR of the model.

Tables 5 and 6 provide the estimates, SE, and OR for contraceptive preference by using a multinomial logistic model. The language variable is constructed by seven dummies, taking Urdu as the reference category. The OR of 1.289 revealed that the modern method is more likely the preferred choice by Pashto speakers compared to Urdu. The OR of the Pashto speakers are approximately the same for natural methods and sterilization (0.980 for natural methods and 0.983 for sterilization) compared to Urdu speakers. Women who speak Saraiki language (OR: 1.185) are more likely to use the natural method of contraception compared to Urdu speakers. Province of the respondent was reconstructed into seven dummies leaving Punjab as the base category. The dummy variable corresponding to KP has positive estimated coefficients for modern methods and sterilized women (0.483 for modern methods and 0.127 for sterilized women) with a standard error of 0.061 and 0.059, respectively, and OR of 1.622 and 1.136, respectively, indicating a higher birth control usage exposure in KPK compared to Punjab. A similar observation is made in respect of Sindh, Islamabad, Azad Jammu Kashmir (AJK), and Gilgit Baltistan (GB). The coefficients of Baluchistan province were observed to be -0.148, -1.081, and -0.285 with standard errors 0.072, 0.136, and 0.067 and OR of 0.862, 0.339, and 0.752 for modern, natural, and sterilized women, respectively. Our results are almost similar to those obtained by Agyei and Migadde [16] and White et al. [36].

### 3.2. Bayesian Logistic and Multinomial Regression Models

The Bayesian model has improved the estimates of sociodemographic factors.  Table 7 shows that the ESS for each coefficient is enough for all coefficients, except Saraiki language in traditional methods, an urban region in sterilization, and the number of children between 1 and 3 in modern methods which are 1674.559, 1483.551, and 1746.864, respectively. This indicates a large enough value to continue with the approach. The ESS for the coefficient of women aged above 44 who are using the birth control method is maximum with 3470.649. The Bayesian logistic regression model predicted that women above 35 years of age have a negative impact on the usage of birth control methods compared to those not using of birth control methods.

Similarly, the estimated coefficient for Khyber Pakhtunkhwa has a positive impact on contraception compared to the Punjab state of Pakistan. We used the Bayesian multinomial logistic regression model for contraceptive methods as a response variable. We specified prior parameters from literature and our knowledge base [28, 35] which is thoroughly discussed in Methods. The function that we are intending to evaluate can be seen by the density plots in the smoothed histograms of the samples. We obtained the trace and density plots, essential for the mixing of chains, for all variables in the MCMC. Figures 3–9 (in the appendix) demonstrate the density and trace plots associated with each model coefficient, providing enough evidence of randomness (lack of pattern) in the data.

The behavior of the posterior density plot for each coefficient is given in the trace plots. Figures 10–19 (in the appendix) show the autocorrelation plots associated with each coefficient and their corresponding lags. Our results reflect those of Maldin and Segal [14].

## 4. Conclusion

We analyzed the birth control behavior of women in Pakistan using two separate models, the classical logistic and multinomial logistic regression model using log-link function, and Bayesian logistic and multinomial regression models. The logistic regression was used to check the behavior of contraception while multinomial logistic regression was used to illustrate the most preferred method of contraceptive use in Pakistan. The analysis executed showed that contraceptive use is almost relevant to sociodemographic factors (education, age, language, partner, work, etc.). Women living in rural areas with low or no education were found to be unaware of contraception. We observed that contraceptive use and methods are most probably influenced by the age and number of children of women [16]. There was a distinctive high significant effect of women on contraceptive use with OR 1.242, 1.155, and 0.633 for women aged 25-34, 35-44, and above 44, respectively, indicating a decrease in OR for contraceptive use as the age of women increases. High-quality education, counseling, and widespread access to contraceptives should be prioritized in family planning healthcare. Women in rural areas of Pakistan are mostly uneducated with a lot of barriers hampering their ability to join school or any formal training to create awareness about themselves. This study can be extended to cover other factors associated with the use of contraceptives used in Pakistan as well as an extended comparison with other countries in the region.

## Figures and Tables

**Figure 1:** Bar graph of contraceptive users across age categories.

**Figure 2:** Multiple bar graph of contraceptive use across provinces and regions.

**Figure 3:** Trace plot 1-A.

**Figure 4:** Trace plot 1-B.

**Figure 5:** Trace plot 1-C.

**Figure 6:** Trace plot 1-D.

**Figure 7:** Trace plot 1-E.

**Figure 8:** Trace plot 1-F.

**Figure 9:** Trace plot 1-G.

**Figure 10:** Autocorrelation of coefficient plot 1-A.

**Figure 11:** Autocorrelation of coefficient plot 1-B.

**Figure 12:** Autocorrelation of coefficient plot 1-C.

**Figure 13:** Autocorrelation of coefficient plot 1-D.

**Figure 14:** Autocorrelation of coefficient plot 1-E.

**Figure 15:** Autocorrelation of coefficient plot 1-F.

**Figure 16:** Autocorrelation of coefficient plot 1-G.

**Figure 17:** Autocorrelation of coefficient plot 1-H.

**Figure 18:** Autocorrelation of coefficient plot 1-I.

**Figure 19:** Autocorrelation of coefficient plot 1-J.

**Table 1:** Variable description.

Variable ID	Variable name	Variable description
V020	EMS	0-never married 1-ever married sample
V213	Pregnant	0-not pregnant 1-pregnant sample
V012	Res_Age	Respondents' age at the time of interview 15 : 49
V024	Province	Province: 1-Punjab, 2-Sindh, 3-KPK, 4-Balochistan, 5-GB, 6-ICT, 7-AJK, 8-FATA
V025	Residence_new	Dummy variable: 0-rural, 1-urban
V701	Edu	Highest educational: 0-no education, 1-primary, 2-secondary, 3-higher
v191	WI	Dummy variable: 1-lower CF, 2-middle CF, 3-high CF
V218	Num_childs	Total children ever born: 1–do not have, 2-among 1 to 3, 3-among 4 to 6, 4-more than 6. v312 contraceptive_method Current contraceptive method 0-not using, 1-pill, 2-IUD, 3-injections, 4-diaphragm, 5-male condom, 6-female sterilization, 7-male sterilization, 8-periodic abstinence, 9-withdrawal, 10-other traditional, 11-implants, norplant 12-prolonged abstinence, 13-lactational amenorrhea (LAM) 14-female condom, 15-foam or jelly, 16-emergency contraception, 17-other modern method, 18-standard days method (SDM), 19-specific method 1, 20-specific method 2, (m) 99-missing Cont_Contraceptive usage Dummy variable: 1-yes, 0-otherwise Cont_Sterilization Dummy variable: 1-yes, 0-otherwise Cont_Modern methods Dummy variable: 1-yes, 0-other Cont_Traditional (natural) Dummy variable: 1-yes, 0-otherwise
V717	Prof_res	“No using” as base category Respondent s occupation (grouped) 0-not working, 1-professional, technical, managerial, 2-clerical, 3-sales, 4-agricultural-elf employed, 5-agricultural-employee, 6-household and domestic, 7-services, 8-skilled manual, 9-unskilled manual, 98-do not know (m) 99-missing
	Prof_tech	Dummy variable: 1-Professional, technical, managerial, or clerical, 0-otherwise
	Prof_Agr	Dummy variable: 1-agricultural-self employed, 0-otherwise
	Prof_Other	Dummy corresponding to remaining categories taking “not working as base”
V045B	Language	lang_interview: 1-English, 2-Urdu, 3-Sindhi, 4-Punjabi, 5-Sariaki, 6-Baluchi, 7-Pushto, 8-otherwise

**Table 2:** Logistic regression of contraceptives used with covariates.

	Estimate	Std. error	OR	Lower CI	Upper CI	Pr (*>*|*z*|)
Intercept	-2.270	0.376	0.103	0.046	0.203	<0.001^∗∗∗^
Age	Reference category “15-24”					
25-34	0.217	0.048	1.242	1.132	1.364	<0.001^∗∗∗^
35-44	0.144	0.049	1.155	1.049	1.273	0.003^∗∗^
Above 44	-0.449	0.054	0.638	0.574	0.710	<0.001^∗∗∗^
Region	Reference category “Urban”					
Urban	0.182	0.024	1.199	1.144	1.257	<0.001^∗∗∗^
Language	Reference category “Urdu”					
Baluchi	-0.785	0.080	0.456	0.390	0.533	0.014^∗∗∗^
English	1.927	1.070	6.866	1.218	128.479	<0.001^∗^
Other	-0.394	0.042	0.675	0.621	0.732	<0.001^∗∗∗^
Punjabi	0.018	0.044	1.018	0.934	1.110	0.682
Pushto	0.044	0.043	1.045	0.961	1.136	0.303
Sariaki	-0.285	0.063	0.752	0.664	0.850	<0.001^∗∗∗^
Sindhi	-0.455	0.051	0.634	0.574	0.701	<0.001^∗∗∗^
Province	Reference category “Punjab”					
AJK	-0.456	0.043	0.634	0.582	0.690	<0.001^∗∗∗^
Balochistan	-0.917	0.053	0.400	0.360	0.443	<0.001^∗∗∗^
FATA	-0.700	0.064	0.496	0.438	0.563	<0.001^∗∗∗^
GB	0.395	0.052	1.484	1.340	1.644	<0.001^∗∗∗^
ICT	-0.063	0.049	0.939	0.854	1.033	0.017
KPK	-0.356	0.046	0.700	0.640	0.767	<0.001^∗∗∗^
Sindh	-0.102	0.050	0.903	0.819	0.996	<0.001^∗^
Education	Reference category “Un-educated”					
Higher	0.294	0.032	1.342	1.260	1.429	<0.001^∗∗∗^
Primary	0.125	0.032	1.134	1.064	1.208	<0.001^∗∗∗^
Secondary	0.124	0.027	1.132	1.073	1.194	<0.001^∗∗∗^
Child	Reference category “Don t have”					
Above 7	2.540	0.374	12.683	6.472	28.686	<0.001^∗∗∗^
Among 1 to 3	1.809	0.373	6.103	3.120	13.784	<0.001^∗∗∗^
Among 4 to 6	2.512	0.374	12.332	6.302	27.861	<0.001^∗∗∗^
Working	Reference category “No”					
Yes	0.198	0.030	1.219	1.151	1.292	<0.001^∗∗∗^
Wealth index	Reference category “Middle class family”					
High class	0.170	0.030	1.185	1.118	1.256	<0.001^∗∗∗^
Low class	-0.485	0.029	0.616	0.581	0.652	<0.001^∗∗∗^

Note: ^∗∗∗^*p* value *<*0.000, ^∗∗^*p* value *<*0.001, ^∗^*p* value *<*0.01, ^+^*p* value *<*0.05, standard error, confidence interval (CI) of the estimates, and odds ratio (OR).

**Table 3:** Regional level logistic regression model of women using contraceptives.

	Rural			Urban			
	Estimate	Std. error	OR	Estimate	Std. error	OR	
Intercept	-2.868^∗∗∗^	0.726	0.057	-1.763^∗∗∗^	0.454	0.172	
Age	Reference category “15-24”						
25-34	0.087	0.067	1.091	0.312^∗∗∗^	0.069	1.366	
35-44	0.047	0.070	1.049	0.192^∗∗^	0.071	1.212	
Above 44	-0.477^∗∗∗^	0.076	0.621	-0.469^∗∗∗^	0.078	0.626	
Language	Reference category “Urdu”						
Baluchi	-0.883^∗∗∗^	0.127	0.413	-0.820^∗∗∗^	0.104	0.440	
English	0.885	1.158	2.422	11.607	98.484	109893.000	
Other	-0.326^∗∗∗^	0.054	0.722	-0.498^∗∗∗^	0.070	0.608	
Punjabi	0.042	0.058	1.043	-0.044	0.074	0.957	
Pushto	0.233^∗∗∗^	0.067	1.263	-0.111^∗^	0.056	0.895	
Sariaki	-0.281^∗∗∗^	0.073	0.755	-0.236	0.161	0.790	
Sindhi	-0.943^∗∗∗^	0.129	0.389	-0.330^∗∗∗^	0.063	0.719	
Province	Reference category “Punjab”						
AJK	-0.549^∗∗∗^	0.062	0.577	-0.378^∗∗∗^	0.061	0.685	
Balochistan	-0.989^∗∗∗^	0.079	0.372	-0.815^∗∗∗^	0.073	0.443	
FATA	-0.963^∗∗∗^	0.093	0.382	-0.339^∗∗∗^	0.099	0.712	
GB	0.439^∗∗∗^	0.069	1.551	0.236^∗∗^	0.085	1.266	
ICT	0.143	0.089	1.153	-0.141^∗^	0.061	0.868	
KPK	-0.501^∗∗∗^	0.073	0.606	-0.263^∗∗∗^	0.061	0.769	
Sindh	0.376^∗∗^	0.128	1.457	-0.156^∗∗^	0.059	0.855	
Education level	Reference category “Un-educated”						
Higher	0.311^∗∗∗^	0.047	1.364	0.256^∗∗∗^	0.046	1.291	
Primary	0.041	0.043	1.042	0.229^∗∗∗^	0.051	1.258	
Secondary	0.170^∗∗∗^	0.036	1.186	0.055	0.042	1.056	
Child	Reference category “Don t have”						
Among 1 to 3	2.455^∗∗∗^	0.724	11.642	1.444^∗∗∗^	0.450	4.238	
Among 4 to 6	3.308^∗∗∗^	0.724	27.338	2.041^∗∗∗^	0.450	7.700	
Above 7	3.376^∗∗∗^	0.724	29.243	1.982^∗∗∗^	0.451	7.256	
Working	Reference category “No”						
Yes	0.158^∗∗∗^	0.041	1.172	0.270^∗∗∗^	0.044	1.309	
Wealth index	Reference category “Middle CF”						
High class	0.109^∗^	0.049	1.116	0.249^∗∗∗^	0.039	1.283
Low class	-0.595^∗∗∗^	0.039	0.552	-0.285^∗∗∗^	0.047	0.752

^∗∗∗^ *p* value *<*0.000, ^∗∗^*p* value *<*0.001, ^∗^*p* value *<*0.01, ^+^*p* value *<*0.05, standard error of the estimates, and odds ratio (OR).

**Table 4:** Province-wise separate logistic regression model of women using contraception.

Balochistan			Sindh		KP		FATA		Punjab		GB		Islamabad		AJK	
Estimate		OR	Estimate	OR	Estimate	OR	Estimate	OR	Estimate	OR	Estimate	OR	Estimate	OR	Estimate	OR
Intercept	-14.130		-13.558		-1.974^∗∗^		-9.885		-1.350^+^		-12.918		0.054		-12.357	
	220.874	0.000	189.351	0.000	0.757	0.139	298.249	0.000	0.760	0.259	266.228	0.000	0.707	1.056	171.800	0.000
Age																
25-34	0.043		0.419^∗∗∗^		0.169		0.718^∗∗∗^		0.2209		0.083				-0.24842	
	0.101	1.043	0.110	1.520	0.108	1.184	0.181	2.050	0.175	1.247	0.176	1.087	0.299^∗^ 0.175	1.348	0.181	0.780
35-44	-0.040		0.305^∗∗^		0.172		0.610^∗∗^		0.209		-0.026		0.285		-0.742^∗∗∗^	
	0.104	0.961	0.114	1.357	0.115	1.188	0.187	1.841	0.185	1.233	0.180	0.974	0.177	1.329	0.200	0.476
Above 44	-0.810^∗∗∗^		-0.264^∗^		-0.299^∗^		0.665^∗∗∗^		-0.0883		-0.793^∗∗∗^		-0.691^∗∗∗^		-1.711^∗∗∗^	
	0.112	0.445	0.124	0.768	0.128	0.741	0.201	1.944	0.203	0.915	0.194	0.452	0.197	0.501	0.236	0.181
Region																
Rural	-0.184^∗^		-0.211^∗∗^		-0.191^∗∗∗^		-0.404^∗∗∗^		-0.213^∗∗∗^		-0.009		0.022		-0.093	
	0.074	0.832	0.066	0.810	0.057	0.826	0.106	0.668	0.051	0.808	0.088	0.991	0.087	1.022	0.066	0.911
Language																
Baluchi	-0.838^∗∗∗^		-14.041													
	0.104	0.433	289.304	0.000												
English	14.180												0.529			
	441.372	1440019											1.160	1.697		
Punjabi	-14.113		0.872^∗^		-0.106				-0.018				-0.186		-0.322	
	624.194	0.528	0.345	2.391	0.095	0.899			0.048	0.982			0.227	0.000	0.241	0.666
Pushto	0.063		1.476^+^		0.761^+^		13.546						-1.378^∗∗^			
	0.099	0.000	0.779	4.374	0.401	2.140	261.723	763736					0.453	0.830		
Sariaki	-0.792^∗∗^		0.487^+^		0.215^∗∗∗^		-0.776^+^		-0.289^∗∗∗^							
	0.293	1.066	0.268	1.628	0.056	1.240	0.430	0.460	0.070	0.749						
Sindhi	-0.261		-0.333^∗∗∗^		-11.774											
	0.167	0.453	0.067	0.717	132.576	0.000										
Other	-0.639^∗∗∗^								-14.955		-0.226^∗∗^		-14.251		-0.407^∗∗∗^	
	0.113	0.771							141.661	0.000	0.073	0.798	239.443	0.252	0.083	0.725
Education level																
Primary	0.670^∗∗∗^		0.420^∗∗∗^		0.211^∗^		0.815^∗∗∗^		0.264^∗∗∗^		0.652^∗∗∗^		0.161		0.142	
	0.127	1.953	0.073	1.522	0.082	1.235	0.167	2.258	0.059	1.302	0.131	1.919	0.112	1.174	0.089	1.153
Secondary	0.974^∗∗∗^		0.478^∗∗∗^		0.733^∗∗∗^		0.414^+^		0.430^∗∗∗^		0.374^∗∗∗^		0.562^∗∗∗^		0.266^∗∗^	
	0.122	2.648	0.079	1.614	0.080	2.082	0.239	1.513	0.067	1.538	0.106	1.454	0.113	1.754	0.085	1.305
Higher	1.355^∗∗∗^		0.684^∗∗∗^		0.948^∗∗∗^		0.255		0.733^∗∗∗^		0.611^∗∗∗^		0.477^∗∗∗^		0.647^∗∗∗^	
	0.172	3.878	0.092	1.982	0.107	2.582	0.347	1.29	0.087	2.080	0.158	1.842	0.115	1.611	0.121	1.909
Number of children																
Among 1 to 3	12.982		13.814		1.737^∗^		11.667		1.994^∗∗^		12.901		0.691		12.781	
	220.874	434698	189.351	998048	0.748	5.679	298.249	116618	0.753	7.347	266.228	400664	0.682	1.995	171.8	355577
Between 4 and 6	13.439		14.692		2.568^∗∗∗^		12.940		3.000^∗∗∗^		13.796		1.267^+^		13.980	
	220.874	686159	189.351	2403132	0.748	13.038	298.249	416685	0.753	20.078	266.228	98103	0.684	3.551	171.800	1178292
More than 7	13.446		14.786		2.656^∗∗∗^		13.666		3.087^∗∗∗^		13.799		0.829		13.623	
	220.874	691119	189.351	2638848	0.750	14.237	298.249	861204	0.756	21.912	266.228	983309	0.693	2.291	171.800	824937
Respondent working																
Yes	-0.262^∗^		0.057		-0.258^∗∗∗^		-0.143		0.166^∗∗^		0.067		0.386^∗∗∗^		0.167^+^	
	0.113	0.770	0.058	1.058	0.094	0.773	0.275	0.867	0.051	1.180	0.155	1.069	0.100	1.472	0.093	1.182
Wealth index																
Poor	-0.337^∗∗∗^		-0.265^∗∗∗^		-0.638^∗∗∗^		-0.665^∗∗∗^		-0.359^∗∗∗^		-0.434^∗∗∗^		-0.034		-0.622^∗∗∗^	
	0.088	0.714	0.079	0.767	0.065	0.528	0.122	0.514	0.059	0.698	0.107	0.648	0.164	0.967	0.080	0.537
Rich	-0.119		0.151^+^		-0.111		0.191		-0.034		-0.284^∗^		-0.022		0.501^∗∗^	
	0.099	0.888	0.077	1.163	0.068	0.895	0.166	1.210	0.059	0.967	0.140	0.753	0.106	0.979	0.081	1.651

Note: ^∗∗∗^*p* value *<*0.000, ^∗∗^*p* value *<*0.001, ^∗^*p* value *<*0.01, ^+^*p* value *<*0.05, standard errors of the estimates are in parenthesis, and odds ratio.

**Table 5:** Multinomial logistic regression model of women with preference of contraception and with covariate effect.

	Modern method			Natural method			Sterilization		
	Estimate	Std. error	OR	Estimate	Std. error	OR	Estimate	Std. error	OR
Intercept	-2.415	0.379	0.089	-10.498	22.309	0.000	-13.378	0.244	0.000
Age									
25-34	0.143	0.057	1.153	0.135	0.068	1.144	2.515	0.321	12.365
35-44	-0.217	0.060	0.805	0.012	0.070	1.012	3.134	0.321	22.957
Above 44	-1.182	0.072	0.307	-0.683	0.078	0.505	2.868	0.322	17.595
Region									
Urban	0.165	0.032	1.179	0.339	0.034	1.404	0.000	0.039	1.000
Language									
English	1.826	1.166	6.209	2.499	1.124	12.168	-5.729	38.548	0.003
Baluchi	-0.268	0.097	0.765	-1.719	0.180	0.179	-1.305	0.175	0.271
Punjabi	-0.136	0.062	0.873	0.099	0.058	1.105	0.049	0.063	1.050
Pushto	0.182	0.054	1.200	0.229	0.060	1.257	-0.783	0.086	0.457
Sariaki	-0.550	0.098	0.577	-0.349	0.091	0.705	-0.022	0.087	0.979
Sindhi	-0.664	0.071	0.515	-1.093	0.078	0.335	0.111	0.073	1.118
Other	-0.378	0.056	0.685	-0.369	0.058	0.691	-0.446	0.076	0.640
Province									
KPK	0.010	0.060	1.010	-0.544	0.064	0.580	-0.749	0.077	0.473
Sindh	-0.008	0.067	0.992	-0.186	0.066	0.830	-0.103	0.073	0.902
Balochistan	-0.637	0.071	0.529	-1.086	0.076	0.338	-1.063	0.089	0.345
GB	0.582	0.068	1.790	0.636	0.067	1.889	-0.452	0.091	0.636
ICT	0.150	0.063	1.162	-0.200	0.065	0.819	-0.168	0.072	0.845
FATA	-0.451	0.083	0.637	-0.728	0.088	0.483	-1.286	0.148	0.276
AJK	-0.350	0.059	0.705	-0.429	0.058	0.651	-0.648	0.067	0.523
Education level									
Primary	0.212	0.045	1.236	-0.008	0.047	0.992	0.145	0.050	1.156
Secondary	0.274	0.037	1.315	0.046	0.038	1.047	-0.016	0.044	0.984
Higher	0.447	0.043	1.564	0.280	0.045	1.323	0.045	0.053	1.046
Number of children									
Among 1 to 3	1.239	0.374	3.452	9.059	22.309	8596	8.708	0.085	6051
Among 4 to 6	1.696	0.375	5.454	9.794	22.309	17933	9.876	0.085	19465
Above 7	1.686	0.376	5.396	9.854	22.309	19036	9.909	0.088	20103
Working									
Yes	0.153	0.041	1.165	0.205	0.042	1.227	0.219	0.042	1.244
Wealth index									
Low class	-0.470	0.039	0.625	-0.430	0.042	0.651	-0.593	0.048	0.552
High class	0.087	0.039	1.091	0.233	0.041	1.262	0.218	0.046	1.244

**Table 6:** Regional level of preference of contraceptive methods and impact of contextual level variables.

	Rural									Urban								
	Modern method			Natural method			Sterilization			Modern method			Natural method			Sterilization		
	Estimate	Std. error	OR	Estimate	Std. error	OR	Estimate	Std. error	OR	Estimate	Std. error	OR	Estimate	Std. error	OR	Estimate	Std. error	OR
Intercept	-3.116	0.730	0.044	-16.423	0.092	0.000	-13.684	0.248	0.001	-1.835	0.457	0.160	-16.764	0.089	0.000	-31.489	0.056	0.000
Age																		
25-34	0.072	0.082	1.075	-0.129	0.099	0.879	1.863	0.324	6.442	0.191	0.080	1.210	0.296	0.095	1.345	14.211	0.046	148499
35-44	-0.315	0.087	0.730	-0.200	0.103	0.819	2.496	0.324	12.130	-0.165	0.084	0.848	0.116	0.098	1.123	14.807	0.036	26954
Above 44	-1.150	0.103	0.317	-0.953	0.115	0.385	2.334	0.326	10.323	-1.263	0.102	0.283	-0.533	0.108	0.587	14.433	0.044	185402
Language																		
Baluchi	-0.855	0.173	0.425	-1.941	0.354	0.144	-0.256	0.208	0.774	-0.096	0.123	0.908	-1.621	0.213	0.198	-13.446	0.000	0.001
English	1.394	1.160	4.031	-14.131	0.001	0.001	-10.725	0.001	0.001	-2.041	0.001	0.130	15.086	0.006	35633	-2.001	0.000	0.135
Other	-0.250	0.071	0.779	-0.245	0.076	0.783	-0.569	0.097	0.566	-0.640	0.099	0.527	-0.464	0.093	0.629	-0.323	0.124	0.724
Punjabi	-0.048	0.081	0.953	0.111	0.079	1.118	0.048	0.082	1.049	-0.339	0.106	0.712	0.101	0.091	1.106	0.011	0.105	1.011
Pushto	0.353	0.085	1.424	0.887	0.113	2.429	-1.127	0.129	0.324	0.013	0.071	1.013	-0.036	0.075	0.965	-0.696	0.118	0.499
Sariaki	-0.512	0.112	0.599	-0.214	0.106	0.807	-0.135	0.105	0.874	-0.767	0.269	0.464	-0.717	0.245	0.488	0.376	0.194	1.456
Sindhi	-1.305	0.172	0.271	-1.149	0.208	0.317	-0.494	0.185	0.610	-0.400	0.087	0.670	-1.160	0.102	0.313	0.311	0.087	1.365
Province																		
AJK	-0.504	0.087	0.604	-0.411	0.087	0.663	-0.759	0.094	0.468	-0.221	0.082	0.802	-0.467	0.080	0.627	-0.509	0.095	0.601
Balochistan	-0.638	0.107	0.528	-1.271	0.125	0.281	-1.384	0.146	0.251	-0.559	0.097	0.572	-1.069	0.101	0.343	-0.797	0.118	0.451
FATA	-0.768	0.121	0.464	-1.370	0.144	0.254	-0.929	0.197	0.395	0.014	0.124	1.014	-0.406	0.128	0.666	-1.348	0.250	0.260
GB	0.628	0.091	1.873	0.675	0.093	1.964	-0.302	0.114	0.739	0.358	0.111	1.431	0.482	0.102	1.620	-0.815	0.165	0.442
ICT	0.319	0.115	1.376	0.096	0.121	1.101	-0.011	0.129	0.989	0.081	0.078	1.084	-0.317	0.079	0.728	-0.213	0.091	0.808
KPK	-0.106	0.095	0.899	-1.222	0.123	0.295	-0.315	0.113	0.730	0.099	0.078	1.104	-0.304	0.078	0.738	-1.031	0.106	0.357
Sindh	0.519	0.167	1.681	0.025	0.200	1.025	0.423	0.182	1.527	-0.080	0.079	0.923	-0.223	0.076	0.800	-0.146	0.087	0.864
Education level																		
Higher	0.469	0.063	1.598	0.214	0.068	1.239	0.190	0.077	1.209	0.387	0.061	1.473	0.334	0.062	1.397	-0.096	0.075	0.908
Primary	0.199	0.060	1.220	-0.086	0.063	0.917	-0.044	0.067	0.957	0.245	0.070	1.277	0.101	0.071	1.107	0.357	0.077	1.429
Secondary	0.337	0.049	1.401	0.027	0.053	1.027	0.085	0.059	1.089	0.180	0.057	1.197	0.059	0.057	1.061	-0.172	0.069	0.842
Number children																		
Above 7	1.947	0.725	7.008	15.110	0.043	36491	9.710	0.090	16476	0.946	0.454	2.576	16.231	0.053	11195	16.213	0.050	10990
Among 1 to 3	2.526	0.725	12.505	16.158	0.044	104097	10.798	0.090	48936	0.828	0.450	2.288	15.560	0.040	57244	15.059	0.052	34678
Among 4 to 6	2.670	0.727	14.436	16.127	0.055	100938	10.906	0.095	54488	1.202	0.450	3.328	16.097	0.041	97935	16.299	0.036	11980
Working																		
Yes	0.033	0.060	1.034	0.115	0.061	1.121	0.299	0.057	1.348	0.281	0.057	1.325	0.318	0.058	1.375	0.179	0.066	1.196
Wealth index																		
High class	0.032	0.065	1.033	0.217	0.068	1.242	0.111	0.074	1.117	0.160	0.051	1.173	0.268	0.053	1.307	0.358	0.063	1.431
Low class	-0.550	0.052	0.577	-0.611	0.056	0.543	-0.637	0.062	0.529	-0.314	0.063	0.731	-0.150	0.066	0.861	-0.461	0.083	0.630

**Table 7:** Bayesian logistic regression and multinomial regression model for using of birth control methods.

	Using contraception			Sterilization			Traditional methods			Modern methods		
	Mean	SD	Eff. size	Mean	SD	Eff. size	Mean	SD	Eff. size	Mean	SD	Eff. size
Intercept	-24.02371	981.64	3000	-24.7646	1021.44	2000	12.84	1006.13	2000	-15.4202	1004.85	2000
Age												
25-34	0.14603	98.98	3111.497	1.18504	99.46	2000	-0.19886	103.81	2178.699	1.2809	98.83	2000
35-44	-2.47666	97.99	3062.794	-2.15375	100.45	2000	-104.716	98.99	2000	0.57232	98.59	2000
Above 44	-2.08556	98.99	3470.649	4.25818	99.66	2146.441	-1.67722	100.14	1870.916	-0.62731	97.5	2296.685
Region (rural)												
Urban	-0.3687	100.74	3000	0.65904	101.27	1483.551	-1.54257	98.36	2000	1.60712	97.72	2000
Province (Punjab)												
Sindh	-0.5241	101.35	3114.08	-1.68469	100.15	2588.433	-0.02649	97.17	2563.114	3.31428	99.47	2000
KPK	1.18738	100.35	3475.173	-1.50089	98.71	1849.171	-0.38554	100.28	2135.33	2.21982	101.19	2000
Baluchistan	-2.26692	99.43	3147.376	-3.45229	101.63	2000	0.86504	97.87	1868.454	3.48583	99.19	2000
GB	-0.56363	97.07	2899.224	2.03009	102.25	2000	-2.39167	100.48	2000	2.98581	101.39	2000
ICT	-2.21406	101.13	2839.384	0.5381	101.67	2000	-3.09084	101.07	2000	-2.47677	101.31	2000
AJK	0.78937	100.81	2845	-2.74986	98.05	2000	1.31417	98.18	2217.355	1.98786	96.93	2000
FATA	3.07512	99.75	3000	4.05026	102.03	2158.799	-1.63813	100.59	2000	0.40811	100.64	2000
Education level (illiterate)												
Primary	-1.54367	100.89	2911.072	0.84124	100.19	2000	4.0359	101.99	2000	-0.23094	103.55	2000
Secondary	1.88213	100.72	2856.31	-0.74852	97.93	2000	-0.53985	102.91	1874.399	0.29983	98.54	2000
Higher	-3.21336	98.97	3116.531	3.91541	101.14	2000	-0.20645	101.49	2175.742	2.02466	99.44	2000
Number of children (do not have)												
BjT (1-3)	0.60203	100.95	3189.979	1.10884	97.45	2000	-1.04728	99.88	2000	0.99706	100.1	1746.864
BjT (4-6)	-1.60033	98.95	2912.802	-6.48082	97.67	2183.979	-2.46676	101.15	2165.103	-2.30453	99.73	2000
Above 7	-1.44049	101.05	3113.793	-1.27317	100.62	2000	1.16778	100.14	2000	-0.29899	102.18	2000
Language (Urdu)												
English	-1.82131	100.39	2902.493	2.0108	100.23	1843.743	-0.23999	100.22	2000	2.93262	99.82	1997.78
Sindh	0.12145	100.27	3107.907	1.48292	99.27	2000	-2.19701	100.18	2000	2.74684	99.5	2000
Punjabi	1.91361	100.85	3244.604	0.44029	97.01	2000	-5.06296	100.89	2217.918	-0.36419	99.83	2000
Saraiki	-0.04503	99.43	3000	1.2694	5 101.32	2000	-0.57013	99.42	1674.559	-2.21593	101.31	2000
Baluchi	3.26365	99.67	3000	-1.90627	98.82	2000	2.92594	99.74	2000	2.07955	97.54	2000
Pashtu	-0.98397	98.36	2834.879	0.63405	99.22	2247.243	-1.45234	102.22	2000	2.0364	99.31	2000
Other	0.12839	100.75	3357.739	-2.56805	99	2000	2.18423	99.09	2000	2.39135	103.18	2000
Wealth index (lower CF)												
Middle CF	-0.35085	99.91	3000	-0.5792	101.42	2000	-0.03552	102.23	2000	-0.26065	99.9	2000
High CF	-1.23766	103.74	3000	-1.39867	100.9	2000	1.48445	99.76	1858.249	-1.06773	98.78	2000
Respondent work (not working)												
Working	-4.53602	100.46	2655.305	2.37891	100.11	2000	-0.07429	98.02	1976.183	2.82451	97.4	1869.782

## Data Availability

The Pakistan Demographic and Health Survey (2017-18) dataset collected by the National Institute of Population Study was used for this study. The data is available at https://www.dhsprogram.com/data/dataset/Pakistan_Standard-DHS_2017.cfm?flag=0.
